# Anterior Segment Optical Coherence Tomography Imaging of Conjunctival Filtering Blebs after Glaucoma Surgery

**DOI:** 10.1155/2014/610623

**Published:** 2014-07-20

**Authors:** Rodolfo Mastropasqua, Vincenzo Fasanella, Luca Agnifili, Claudia Curcio, Marco Ciancaglini, Leonardo Mastropasqua

**Affiliations:** ^1^Ophthalmology Unit, Department of Neurological, Neuropsychological, Morphological and Movement Sciences, University of Verona, 53593 Verona, Italy; ^2^Ophthalmic Clinic, Department of Medicine and Aging Science, Ophthalmic Clinic, University G. d'Annunzio of Chieti-Pescara, Via dei Frentani 114, 66100 Chieti, Italy; ^3^Excellence Eye Research Center, CeSI, G. d'Annunzio University of Chieti-Pescara, 66100 Chieti, Italy; ^4^Ophthalmic Clinic, Department of Surgical Science, University of L'Aquila, 67100 L'Aquila, Italy

## Abstract

Time domain (TD) and spectral domain (SD) optical coherence tomography (OCT) are cross-sectional, noncontact, high-resolution diagnostic modalities for posterior and anterior segment (AS) imaging. The AS-OCT provides tomographic imaging of the cornea, iris, lens, and anterior chamber (AC) angle in several ophthalmic diseases. In glaucoma, AS-OCT is utilized to evaluate the morphology of AS structures involved in the pathogenesis of the disease, to obtain morphometric measures of the AC, to evaluate the suitability for laser or surgical approaches, and to assess modifications after treatment. In patients undergoing surgery, AS-OCT is crucial in the evaluation of the filtering bleb functionality, permitting a combined qualitative and quantitative analysis. In this field, AS-OCT may help clinicians in distinguishing between functioning and nonfunctioning blebs by classifying their macroscopic morphology, describing bleb-wall features, bleb cavity, and scleral opening. This information is critical in recognizing signs of filtration failure earlier than the clinical approach and in planning the appropriate timing for management procedures in failing blebs. In this review, we summarize the applications of AS-OCT in the conjunctival bleb assessment.

## 1. Introduction

The only treatment of proven efficacy in glaucoma is still the reduction of intraocular pressure (IOP) [1]. However, several patients do not achieve the required target IOP despite maximum tolerated medical therapy or may become intolerant to medication because of adverse events thus reducing compliance [2]. In these cases, a surgical approach is warranted in order to control IOP and reduce the rate of damage progression [3]. Surgical filtration procedures for glaucoma may be classified as either penetrating or nonpenetrating, depending on the removal or preservation of the trabeculo-Descemet membrane, respectively. Trabeculectomy represents the most common and effective penetrating surgical procedure for glaucoma and is still the gold standard surgery. Deep sclerectomy and viscocanalostomy were proposed as nonpenetrating filtration procedures, with the aim of reducing the occurrence of postoperative complications [4]. All filtration procedures lead to an elevation of the conjunctiva at the site of surgery, which is commonly referred to as a filtering bleb. A filtering bleb is considered a cornerstone of IOP control after glaucoma filtration surgery [5–8] and, to a lesser degree, after drainage device implantation. This critical structure allows aqueous humor (AH) to drain from the anterior chamber (AC) into the subconjunctiva, lowering the IOP. However, in a significant number of cases AH filtration fails [9] subsequent to conjunctival fibrosis within the bleb wall.

New imaging diagnostic methods such as anterior segment-optical coherence tomography (AS-OCT) [10] and in vivo laser scanning confocal microscopy (LSCM) [11–15] can be used in conjunction with clinical evaluation to assess morphology and function of blebs and to distinguish functioning from nonfunctioning blebs. These techniques can identify precocious signs of conjunctival fibrosis prior to identification with clinical assessment.

The aim of this review was to summarize the application of the AS-OCT on morphofunctional assessment of conjunctival filtering blebs after glaucoma surgery.

## 2. Methods of Literature Search

PubMed searches were performed on April 22, 2014, using the phrases “anterior segment-optical coherence tomography or AS-OCT and blebs,” “anterior segment-optical coherence tomography or AS-OCT and glaucoma filtration surgery,” and “filtering blebs and anterior segment-optical coherence tomography or AS-OCT” for publications from 1980 to April 2014. Articles in English were fully reviewed; articles in other languages were reviewed using their English abstracts when available.

## 3. Platforms and Technical Characteristics of the AS-OCT

AS-OCT is a noncontact method that provides cross-sectional, three-dimensional, high-resolution images of the anterior segment of the eye, with an axial resolution ranging from 3 to 20 *μ*m. It provides qualitative and quantitative assessment of the most important structures involved in the pathogenesis of glaucoma, such as those defining the iridocorneal angle. Moreover, AS-OCT is used to evaluate anatomical variations of these structures after glaucoma surgery to determine the position of tubes within the AC and to assess bleb features and functionality.

Two OCT platforms are currently available: time domain (TD-OCT) and spectral domain (SD-OCT). The most diffuse and studied anterior segment TD-OCT for glaucoma is the Visante OCT (Carl Zeiss Meditec, Inc., Dublin, CA). Visante has a scanning speed of 4,000 axial scans per image and image acquisition rate of 8 frames/sec with an axial resolution of 18 *μ*m and a lateral resolution of 60 *μ*m.

SD-OCT systems include the RTVue (Optovue, Inc., CA), the Cirrus (Carl Zeiss Meditec), the Spectralis (Heidelberg Engineering, Inc.), and the Casia SS-1000 OCT (Tomey, Nagoya, Japan) [17]. SD-OCT platforms have several advantages over TD-OCT. First, this imaging modality yields high-resolution images that are almost similar to those obtainable with histological preparations. Second, in SD-OCT the scanning speed is much higher than in TD-OCT (ranging from 26.000 to 40.000 A-scans per second); thus, measurement time and overall exam duration are reduced, with better patient comfort. Third, SD-OCT platforms assess both the posterior and anterior pole of the eye (with the cornea/anterior segment modules). Finally, dedicated software permits a three-dimensional assessment of AC structures and conjunctival bleb.

On the other hand, the optical cross-sections obtained with SD-OCT have less tissue penetration than TD-OCT. Therefore, while SD-OCT is able to show features of the bleb wall such as the optically empty cystic spaces and scarring processes, this imaging technique is less adapt in imaging deep structures such as the scleral flap, intrascleral lake, and internal ostium [18] (Figure 1).

## 4. AS-OCT of Filtering Blebs after Penetrating Filtration Surgery

### 4.1. Trabeculectomy

The macroscopic appearance and the microscopic features of conjunctival blebs have predictive implications for surgical outcomes of trabeculectomy. The clinical evaluation of the filtering ability of a bleb incorporates well-established parameters such as the extent, elevation, and vascularity of the conjunctiva at the site of surgery. Unfortunately, in some cases, there is no correlation between the bleb appearance and the IOP. This can lead to difficulty in assessing the filtering ability with slit-lamp evaluation and in recognizing the signs of failure in time.

Different bleb classification systems were proposed [19–21]. According to these systems, a functioning bleb presents a diffuse or cystic shape, with a mild elevation over the scleral flap, few conjunctival vessels, and evidence of microcysts within the conjunctival epithelium. On the other hand, failed blebs are characterized by a small superficial extension without elevation at the site of surgery (flat shape) or with a high degree of elevation with excessive and irregular vascularization (encapsulated shape). However, these systems present some limitations such as assignment of a single vascularity grading and coarse grading scales and are unable to describe blebs with mixed morphology. Currently, the most used grading systems, which for the most part overcome these limitations, are the Moorfields bleb grading system (MBGS) and the Indiana bleb appearance grading scale (IBAGS) [22]. The MBGS defines the bleb functionality by considering the area, height, and vascularity, whereas the IBAGS considers also the AH leakage with Seidel test.

Wells et al. [23] reported that both systems performed adequately in defining the bleb morphology, were clinically reproducible, and had generally high levels of interobserver agreement. MBGS performed similarly to the IBAGS for reproducibility, had higher intraclass correlation coefficient values for morphologic characteristics, and captured extra vascularity data. However, both systems presented minor deficiencies with possible loss of information.

In cases in which slit-lamp examination cannot provide clear and complete information, advanced imaging technologies may help clinicians in defining the exact morphological bleb type and in differentiating between functioning from failing or failed blebs.

LSCM was used to study the conjunctiva before and after different surgical and medical therapies for glaucoma to analyze AH outflow pathways modifications [16, 24–26]. In filtration surgery, LSCM proved valuable in assessing the drainage capability of conjunctival blebs by assessing microcysts density and area within the epithelium, and the collagen deposition within the stroma [12–15]. While LSCM permits a microscopic analysis, with the advantage of analyzing tissue at a cellular level, AS-OCT allows a macroscopic analysis, useful to classify blebs according to their morphology.

Several studies have analyzed if TD-OCT (Visante OCT) can be used to distinguish between functioning and nonfunctioning filtering blebs [27, 28]. Leung et al. [27] differentiated blebs according to their global appearance: diffuse or cystic blebs were classified as functioning, whereas encapsulated or flattened blebs were classified as nonfunctioning. Additionally, while functioning blebs presented a low to medium reflectivity of the external wall with a wide inner fluid-filled cavity, failed blebs presented with opposite features (Figures 2 and 3). Pfenninger et al. [29] reported a significant direct correlation between the reflectivity of the fluid-filled cavity and the IOP, whereas Tominaga et al. [30] found a significant inverse correlation between the bleb-wall thickness and IOP. On the contrary, the same authors did not find significant correlation between the height and extent of the filtering bleb cavity and the IOP.

Generally, AS-OCT features are in agreement with microscopic findings as seen with LSCM: in functioning trabeculectomy, the bleb wall appears low reflective and thick at AS-OCT, with numerous intraepithelial microcysts and a loosely arranged stroma at LSCM. Conversely, failed blebs show the opposite features (Figures 2 and 3) [12]. Ciancaglini et al., [12] in a study that proposed a combined clinical and instrumental approach to evaluate the filtering bleb functionality, found a good degree of concordance between the clinical and AS-OCT bleb classification, particularly for the cystic (100%) and diffuse (74%) patterns. Thus, AS-OCT may support clinicians in correctly classifying blebs. In the same study, the use of MMC produced a significantly higher mean longitudinal radial length, indicative of a diffuse functioning bleb, compared to eyes that had not received antimetabolites.

The introduction of SD-OCT yielded obtaining additional or more defined information of the bleb morphology. Kawana et al. [31] studied the internal structures of blebs after trabeculectomy using a 3-dimensional cornea AS-OCT (3-D CAS OCT) reporting that AH intrableb drainage routes, bleb-wall microcysts, and the scleral flap could be visualized in more than 90% of the cases. Successful blebs presented a large internal fluid-filled cavity, a wide hyporeflective area, and thicker walls with a higher number of microcysts. The 3D AS-OCT proved valuable also in identifying the exact filtration openings after trabeculectomy, where AH flows through the sclera into the bleb cavity [32]. Particularly, filtration openings were identified in the 95% of cases and were mostly located in the middle third of the scleral flap margins; moreover, 24% of blebs presented two or more scleral openings.

### 4.2. Ex-PRESS Implant

AS-OCT also provides high-resolution imaging in eyes implanted with glaucoma drainage devices, helping clinicians in identifying the position and patency of tubes in AC, AH outflow pathways, and the occurrence of complications such as corneal- or iris-tube contact. The Ex-PRESS glaucoma filtration device (Alcon Laboratories, Fort Worth, Texas, USA) is a small stainless steel, nonvalved, MRI-compatible implant (available with a 50 or 200 *μ*m lumen). It lowers IOP by shunting AH from the AC into the subconjunctiva, creating a bleb similar to that produced by trabeculectomy. The procedure, in fact, is an alternative to trabeculectomy. Very recently, the XTV study [33] reported that mean IOP, medication use, and surgical success were similar at 2 years after EX-PRESS implantation or trabeculectomy, with fewer complications in eyes that received the Ex-PRESS device. Verbraak et al. [34] used an experimental AS-OCT to evaluate porcine eye after Ex-PRESS implantation ex vivo, clearly visualizing the entire outline and position of the implant. However, to date, studies that evaluated filtering blebs characteristics in human eyes implanted with Ex-PRESS, and studies that analyzed differences in bleb morphology after trabeculectomy or Ex-PRESS implantation, are still lacking.

It can be hypothesized that blebs after Ex-PRESS implantation present some morphological differences with respect to blebs after trabeculectomy since the AH flows through artificial scleral channels with different lumen sizes and morphology. In the case of Ex-PRESS implant, a regular tube creates the scleral channel; in trabeculectomy, a transscleral channel extending from the position formerly occupied by trabecular meshwork to the subconjunctiva is formed. The channel formed following trabeculectomy is irregular, since it is a network of extended fibroblasts with loosely arranged collagenous tissue and a large number of vessels [35]. Thus, the difference in hydrodynamic effects that AH undergoes in order to reach the subconjunctival space may lead to a different modulation and a final different shape of the bleb.

In large case series of patients implanted with Ex-PRESS (P200 model)/MMC or who underwent trabeculectomy/MMC (unpublished data), we observed with SD-OCT (RTVue, Optovue, Inc., CA) that blebs after Ex-PRESS implants presented a diffuse shape, with a uniform and posteriorly directed AH filtration, probably expression of a regulated AH passage toward the subconjunctiva (Figure 4(a)). Conversely, filtering blebs derived from trabeculectomy were more commonly cystic with a less extended (even though higher) subconjunctival area, probably expression of a more turbulent AH passage toward the subconjunctiva (Figure 4(b)). On this basis, further structured studies assessing bleb morphology with AS-OCT in patients undergoing trabeculectomy or Ex-PRESS device are warranted.

Also the position of the device, in relation to the limbal margin, may have a significant effect on bleb morphology and final surgical success. In the same case, series blebs showed a smaller subconjunctival area, a hyperreflective wall with a flat shape (Figure 5(a)) when the device was placed anteriorly (arrowhead, 0 to 1 mm from the limbus). Oppositely, a higher subconjunctival filtration area, a lower reflective wall, and a more diffuse or cystic shape were evident when Ex-PRESS was implanted more posteriorly in the scleral bed (1 to 2 mm from the limbus) (Figure 5(b)) (RTVue, Optovue, Inc., CA). When comparing the overall surgical success (six-month follow-up, one third reduction of IOP from baseline), the Ex-PRESS devices implanted posteriorly presented a significantly higher success rate compared to devices implanted anteriorly (75% versus 38%; *P* < 0.001). By hypothesizing, this could be due to the fact that a device implanted too anteriorly do not allow a useful posterior AH outflow, which is critical to promote the formation of a diffuse and functioning filtering bleb.

## 5. AS-OCT of Conjunctival Bleb in Nonpenetrating Filtration Surgery

Nonpenetrating filtration surgery was proposed as an alternative to trabeculectomy with the aim of reducing intra- and postoperative complications [36]. Nonpenetrating deep sclerectomy and viscocanalostomy, which have now abandoned the clinical scenario, were the two proposed nonpenetrating procedures. Aptel et al. [37] used the AS-OCT to study filtering blebs after deep sclerectomy with collagen implant, reporting that lower IOP values correlated with a thinner and lower reflective bleb wall and with larger subconjunctival fluid spaces.

## 6. AS-OCT of Filtering Blebs after Glaucoma Drainage Device Implantation

In a recent study, [38] Jung et al. reported that Visante OCT proved valuable in the morphological assessment of blebs in patients who underwent Ahmed glaucoma valve (AGV) implantation. The authors observed a significantly lower maximum bleb-wall thickness in successful compared to unsuccessful AGV implants. This aspect, which was the opposite to that found in filtering blebs of successful trabeculectomy, could be determined by the presence of silicone drainage device, which impedes direct absorption of AH by the conjunctiva. Moreover, AS-OCT did not identify microcysts and collections of multiloculated fluid cavities within the bleb wall above the plate of the valves, which, conversely, are common in trabeculectomy [27, 31]. No significant differences were found between successful and failed AGV concerning the bleb-wall reflectivity, which presented a high signal in all cases. Therefore, the bleb morphology above the drainage valve plate was quite similar to that of encapsulated blebs after unsuccessful filtration surgery with a fluid-filled space surrounded by a connective tissue with a high reflectivity [27]. Therefore, conjunctiva blebs after glaucoma valve are morphologically different from blebs formed after filtration surgery, suggesting that AH reabsorption is only in part linked to the bleb drainage ability.

## 7. AS-OCT in the Bleb Management Procedures

The early postoperative period represents the most critical period for the bleb survival and the long-term surgical success. Frequently, several procedures are required to reduce the scarring processes and maintain an effective AH filtration through the scleral flap margins and the layers of conjunctival bleb wall. Various procedures may be adopted to preserve the bleb functionality. The AS-OCT could be a useful tool to support the decision-making process for the timing and choice of the most appropriate procedure to adopt in failing blebs.

*Finger Massage.* Finger massage is a common technique employed after filtering surgery to aid the AH flow through the artificially created pathway. This procedure promotes the patency of the scleral channel, with the subsequent expansion of the subconjunctival space. Bulbar massage can be done with fingers or with an ocular massage device. In a pilot study, Gouws et al. [39] compared these two techniques but did not find a statistically significant difference in terms of IOP between methods. On the other hand, the use of the device presented a greater ease of use and lower pain scores.

No previous studies were conducted on the application of AS-OCT for studying bleb modifications before and after bulbar massage. In a prospective case series study (unpublished data) conducted with SD-OCT (RTVue, Optovue, Inc., CA), we evaluated the modification of the fluid-filled cavity area, bleb-wall thickness, and scleral opening before and after bulbar digital massage (60 seconds of duration). We observed a significant decrease of IOP with an increase of the bleb-wall thickness, intraepithelial microcysts, and the fluid-filled cavity area more extended posteriorly (Figure 6). Of note, all these variables returned to baseline values after 120 minutes.

*Subconjunctival Injections of Antimetabolites. *To date, studies on the application of AS-OCT after subconjunctival antimetabolites injections are not available. Our group recently conducted a prospective randomized, double blind, six-month study (unpublished data, currently under peer review) to compare the long-term effect of peribleb injection of 5-fluorouracil (5-FU; three weekly injections for three weeks) versus phosphate buffered solution (PBS; three weekly injections for three weeks) in patients with failing blebs (progressive IOP increase in the last two weeks, flattening or encapsulation of the conjunctiva at slit lamp, decrease of the density of intraepithelial microcysts and stromal scarring at LSCM, bleb-wall hyper-reflectivity at AS-OCT). In blebs injected with 5-FU the SD-OCT (RTVue, Optovue, Inc., CA) showed a less reflective and thicker bleb wall, with multiple intra- and subepithelial fluid filled cavities, compared to eyes treated with PBS (Figure 7).

*Bleb Needling. *The bleb-wall fibrosis is the more common long-term complication and the first cause of failure of filtration surgery. In addition, the intra- and episcleral fibrosis is also involved in the final blockage of the AH outflow. The needling procedure is aimed at mechanically removing the connective capsule under the bleb wall and the fibrotic adhesion in the bleb cavity in failing encapsulated blebs, by using a needle. During procedure, a needle is moved in a side-to-side motion, breaking episcleral adhesions over the scleral flap and within the bleb cavity. To improve the efficacy of the bleb needling, revisions with 5-FU were proposed by Ewing and Stamper [40]. Guthoff et al. [41] analyzed the bleb modifications with AS-OCT before and after needling, reporting a collapse of the intrableb cysts in five patients out of nine; notably, only those patients in whom cysts collapsed presented a controlled IOP without glaucoma medication after six months.

*Laser Suture Lysis (LSL). *In a prospective observational case series study Singh et al. [42] reported that AS-OCT significantly affected the decision-making process concerning LSL after trabeculectomy. In this study, LSL was recommended in 100.0% of cases based on clinical findings of elevated IOP, deep AC, and a poorly formed bleb. When AS-OCT was used to decide whether to perform LSL or not, this procedure was recommended in 71.4% of cases, particularly in blebs showing opposed scleral flaps, absent subflap spaces, and thin bleb wall. Moreover, AS-OCT can also be used to assess bleb modifications after LSL. In successful treatments, a separation of the scleral flap from the scleral bed is evident (Figure 8), with facilitation of the AH drainage and the elevation of the conjunctiva at the site of bleb [43, 44]. 

*Filling Implants. *The insertion of filling implants within the bleb or the scleral lake may be considered as an intraoperative bleb management procedure, aimed at reducing the rate of failure after penetrating or nonpenetrating filtration surgery. In penetrating surgery, these implants act as space maintainers between the scleral flap and conjunctiva in the early postoperative period, facilitating the AH passage through the conjunctival layers, and limiting fibrotic processes. In addition, such implants reduce the incidence of hypotony, acting as mechanical compressors over the scleral flap. In nonpenetrating surgery, filling implants also promote the preservation of the intrascleral lake. Space filling implants can be differentiated in absorbable and nonabsorbable. The HEALA flow (a slowly absorbable viscoelastic implant), the SK-gel (SKGEL 3.5 (Corneal Laboratories, Paris, France); sodium hyaluronate implant), and the Ologen (a disc-shaped porcine-derived biodegradable collagen matrix) are absorbable implants. The T-flux (T-Flux device; IOLTECH Laboratories, La Rochelle, France) used during deep sclerectomy is nonabsorbable.

To date, their utility is still controversial [45, 46]. In a prospective randomized trial Cillino et al. [47] compared the Ologen implant as adjuvant versus low-dosage MMC in trabeculectomy and used AS SD-OCT (Topcon 3DOCT-1000, Topcon Corporation, Tokyo, Japan) to evaluate bleb morphology. The authors reported that SD-OCT did not show qualitative differences in the bleb-wall appearance between groups, indicating that the Ologen implant did not enhance or modify the morphology of the bleb wall. Nevertheless, SD-OCT documented a thicker bleb wall in successful Ologen-augmented trabeculectomy with respect to MMC-augmented successful trabeculectomy. In consistence with these results, in our case series (unpublished data) Optovue did not document significant differences of bleb morphology in patients implanted with Ologen compared to patients who did not receive the device (Figure 9).

## 8. Limitations

One of the shortcomings of AS-OCT in assessing filtering blebs is that it does not provide microscopic information (as all imaging modalities), which is essential for detecting the very early signs of failure, such as the stromal collagen deposition and the reduction of AH filled epithelial microcysts. Moreover, features indicative of bleb inflammation (dendritic cell activation and lymphocyte infiltration) or infection (infiltration of mononucleate inflammatory cells) cannot be detected. Therefore, AS-OCT may probably identify failing blebs in a later time with respect to microscopic methods of analysis such as LSCM. Further prospective studies evaluating the ability of these methods in detecting the early signs of failure over time are warranted.

## 9. Discussion and Conclusion

The main challenge in the management of filtration surgery is the preservation of the AH outflow through the scleral ostium and the bleb in order to maintain a good IOP control. Therefore, a careful postoperative clinical evaluation is strongly recommended because the bleb filtering ability may decrease over time. In several cases, the slit-lamp appearance may not be indicative of the bleb functionality because the clinical analysis is a qualitative assessment affected by the intra- and interobservers variability. In addition, the presence of collagen fibers within the bleb wall, especially in cases of florid connective deposition, may impede the visualization of the deeper layers of the bleb wall, the inner cavity, and the scleral flap. Therefore, clinical assessment cannot permit a timely identification of signs of filtration failure.

AS-OCT may contribute to overcome these problems by allowing a detailed structural assessment of bleb-wall layers, bleb cavity, and scleral opening. Moreover, this methodology provides essential biometric parameters such as the bleb-wall reflectivity and thickness, the inner cavity diameters and area, which may help the clinician in distinguishing between functioning from nonfunctioning blebs. In addition, AS-OCT proved valuable in the early identification of signs of failure, critical for the bleb management. This is essential to preserve AH filtration since bleb management procedures are much more effective when administered very early. Therefore, a postsurgical follow-up that also considers the routinely use of AS-OCT with the clinical evaluation is recommended in order to obtain detailed information concerning bleb functionality.

In closing, a combined diagnostic approach that comprehends the standard clinical evaluation and an imaging technique such the AS-OCT may improve the clinician's ability in the understanding bleb functionality, in planning the correct timing for bleb management procedures, and in the evaluation of their efficacy.

## Figures and Tables

**Figure 1:** Spectral domain- (SD-) and time domain- (TD-) OCT assessment of a cystic filtering bleb. Slit-lamp biomicroscopy of a functioning cystic bleb after Ex-PRESS implant (a and b). Bleb images (taken at the same point) as obtained with SD-OCT (Optovue and Spectralis, resp.) (c and d) and TD-OCT (Visante OCT) (e). SD-OCT presents a higher resolution with a more detailed visualization of bleb-wall layers, inner cystic spaces, and the limit between scleral bed and bleb, with respect to TD-OCT. On the other hand, SD platforms seem to have less tissue penetration than TD- OCT (arrows).

**Figure 2:** Functioning filtering blebs. Functioning blebs, after MMC-augmented trabeculectomy, present a diffuse (a) or a cystic shape (b) at clinical evaluation. At AS-OCT (Visante OCT) these blebs show a patent and low reflective inner cavity (asterisks) (c and d), multilobed in the cystic shape, and a thick and low reflective bleb wall. In vivo laser scanning confocal microscopy (e) shows numerous intraepithelial microcysts in a glaucomatous patient after successful MMC-augmented trabeculectomy (planar reconstruction of the superior bulbar conjunctiva 6 weeks after surgery). (e: from Ciancaglini et al., [15] with permission from the publisher).

**Figure 3:** Failed filtering blebs. Nonfunctioning blebs, after MMC-augmented trabeculectomy, appear flat (a) or encapsulated (b) at clinical evaluation. At AS-OCT (Visante OCT) (c and d) these blebs present a patent and low reflective inner cavity but with a thick and hyperreflective bleb wall (arrows). In vivo laser scanning confocal microscopy (e) shows scattered and markedly less numerous intraepithelial microcysts in a glaucomatous patient who underwent failed MMC-augmented trabeculectomy (planar reconstruction of the superior bulbar conjunctiva 6 weeks after surgery). Arrowhead indicates the Ex-PRESS implantation. (e: from Mastropasqua et al., [16] with permission from the publisher).

**Figure 4:** Filtering bleb features after trabeculectomy and Ex-PRESS implantation. Conjunctival filtering bleb after successful MMC/Ex-PRESS (P200) implantation (arrowhead) (a) shows a uniform and regular diffuse pattern, with AH drainage well extended posteriorly to the scleral flap. Differently, bleb after MMC/trabeculectomy (b) presents a cystic pattern with a less regular shape (RTVue, Optovue, Inc, CA).

**Figure 5:** Filtering bleb features after Ex-PRESS implantation according to the position of the device. Bleb morphology may be significantly affected by the position of the device within the scleral bed. In anteriorly positioned Ex-PRESS implant (a) (0-1 mm from the limbal margin (L); arrowhead), the bleb presents features of a failed filtration, with a flat shape (asterisk), limited subconjunctival area (scattered cysts), and a hyperreflective bleb wall. Conversely, in posteriorly positioned Ex-PRESS implant (b) (1 to 2-3 mm from the limbal margin (L); arrowhead), the bleb presents features of an effective filtration, with a cystic multilobed shape (asterisk), a wide subconjunctival filtration area, and a low reflective bleb wall (RTVue, Optovue, Inc, CA).

**Figure 6:** Effects of the digital ocular massage on filtering bleb morphology. Sixty seconds after bulbar digital massage of an eye implanted with Ex-PRESS (arrowhead), the fluid-filled cavity area extended posteriorly (asterisks), bleb-wall thickness increased, and several intraepithelial cysts appeared (arrows) compared to baseline (b and a, resp.) (RTVue, Optovue, Inc, CA).

**Figure 7:** Effects of 5-FU injections on filtering bleb morphology. Blebs injected with subconjunctival 5-FU (extrableb injection) showed a less reflective and thicker bleb wall, with multiple intra- and subepithelial fluid filled cavities (b), compared to eyes treated with PBS, which presented opposite signs without evidence of filtration (a). Arrowhead represents Ex-PRESS device (RTVue, Optovue, Inc, CA).

**Figure 8:** Filtering bleb morphology modifications after laser suture lysis (LSL). Nonfunctioning encapsulated filtering bleb (a) showing a subconjunctival fluid filled cavity isolated from the anterior chamber because of the tight contact of the flap with the surrounding sclera. After LSL the scleral flap appears separated from the surrounding sclera, with restoration of the access (asterisk) with the anterior chamber (b) (Visante OCT).

**Figure 9:** Filtering bleb morphology after biodegradable collagen matrix implantation. Three months after the subconjunctival implantation of the Ologen (a), no significant morphological differences in the macroscopic bleb structure are evident (except for a thicker bleb wall) compared to eyes that did not receive the implant (b).
